The article "Gambogic Acid and Piperine Synergistically Induce Apoptosis in Human Cholangiocarcinoma Cell via Caspase and Mitochondria-Mediated Pathway" was published in 2022. Journal: Evid Based Complement Alternat Med.

# Gambogic Acid and Piperine Synergistically Induce Apoptosis in Human Cholangiocarcinoma Cell via Caspase and Mitochondria-Mediated Pathway

**DOI:** 10.1155/2022/6288742

**Published:** 2022-05-12

**Authors:** Rittibet Yapasert, Ratana Banjerdpongchai

**Affiliations:** ^1^Department of Biochemistry, Faculty of Medicine, Chiang Mai University, Chiang Mai 50200, Thailand; ^2^Center for Research and Development of Natural Products for Health, Chiang Mai University, Chiang Mai 50200, Thailand

## Abstract

Most cholangiocarcinoma (CCA) patients undergo chemotherapy as a therapeutic approach due to the disease's frequently late diagnosis. However, because CCA is resistant to currently available treatments, the prognosis for this cancer is still quite poor. Combination therapy has emerged as a novel and promising strategy in cancer treatment, as monotherapy frequently results in tumor recurrence and drug resistance. Gambogic acid has been shown to have a synergism with other compounds in combating certain cancer cells. Moreover, piperine has been shown to improve the efficacy of numerous chemotherapy drugs and other anticancer natural substances. However, no research has been done on the combination of these two compounds in the treatment of bile duct cancer. In this study, the cytotoxic activity was determined by using the MTT assay, and then, the combined effect was assessed by using the combination index (CI). We found that the combination of gambogic acid and piperine inhibited cell viability more effectively than either treatment alone, and it also demonstrated a synergistically cytotoxic effect against CCA cells. Interestingly, the findings allowed the use of lower concentrations of gambogic acid in cancer treatment when combined with piperine, which could reduce its adverse effect on normal cholangiocytes. Furthermore, the combination of the two compounds increased CCA cell death by inducing apoptosis via both the extrinsic and intrinsic or mitochondria-mediated pathways, as determined by caspase-3, -8, and -9 activity and the reduction of mitochondrial transmembrane potential (ΔΨm). It is possible that the use of these two natural compounds together could be a promising strategy for the treatment of bile duct cancer.

## 1. Introduction

Primary hepatic cancer, often known as liver cancer, is classified into two histopathological types: hepatocellular carcinoma (HCC) and cholangiocarcinoma (CCA). HCC is the most frequent type of liver cancer around the world [1]. CCA is highly prevalent in Thailand and is the most common pathogenic form, accounting for more than 80% of all detected primary liver cancer [2, 3]. CCA is still associated with high mortality rates, particularly in the northeast of Thailand, due to its aggressiveness and the poor prognosis generally in patients suffering from this disease [1, 4, 5]. At present, only about a quarter of CCA patients are candidates for surgical excision of the tumor, with the majority of the patients undergoing chemotherapy as a type of treatment [6]. Unfortunately, CCA cannot resist standard treatment by using several tolerance pathways [7, 8]. As a result, it is critical to find a novel drug with great efficacy for CCA treatment [9, 10].

Gambogic acid (see Figure 1(a)) is the major xanthonoid derived from the brownish resin of the *Garcinia hanburyi* tree in Southeast Asia [11, 12]. Previous studies have revealed its anticancer efficacy both *in vitro* and *in vivo*. In preclinical research, the cytotoxicity and the effect on apoptosis induction of gambogic acid were demonstrated. Gambogic acid can inhibit HCC and CCA cell proliferation, induce cell cycle arrest at the G0/G1 phase, and then induce apoptosis through both the mitochondria-dependent and extrinsic death receptor pathways [13–16]. However, in animal studies, this compound has been shown to cause a variety of adverse effects as well as severe systemic toxicity [17–20].

Piperine (see Figure 1(b)) is a major alkaloid isolated from *Piper nigrum* (black pepper) and *Piper longum L*. (long pepper) [21], both of which are used in culinary and traditional medicine around the world. Piperine has several pharmacological effects, including anticonvulsant [22], antioxidant [23], antiinflammatory [24], antiangiogenic [25], antibacterial [26], and anticancer activities. It has been shown in recent research to be cytotoxic to a variety of human cancer cells [27–29]. Furthermore, piperine can induce mitochondria-mediated apoptosis in HCC cells [30]. These findings imply that it may have a therapeutic potential against CCA. Intriguingly, it is a known bioavailability enhancer for various chemotherapeutic agents and other anticancer natural compounds because of its inhibitory effect on p-glycoprotein or multidrug resistance protein 1 (MDR1) activity [31, 32].

Monotherapy frequently results in tumor recurrence and drug resistance [33], whereas combination therapy has emerged as a novel and promising strategy in cancer treatment [34, 35]. Given their similar killing mechanisms, we intended to test whether these two natural chemicals when combined have greater anticancer potential while having fewer negative effects on normal cells (cholangiocytes). In the present study, we examined the effects of gambogic acid and piperine alone or in combination on CCA cell proliferation and apoptosis. Our studies demonstrated that cotreatment of gambogic acid with piperine enhanced the cytotoxic effect and apoptosis in CCA cells, while decreasing toxicity in normal cholangiocytes when compared to a single compound treatment, suggesting that the combination of these two compounds may deliver a novel and advantageous option for treatment of CCA patients.

## 2. Materials and Methods

### 2.1. Chemical Compounds

Gambogic acid (purity ≥ 95%) was purchased from Cayman Chemical (2752-65-0) (Ann Arbor, MI, USA). Piperine (P49007) (purity ≥9 7%) and gemcitabine (G6423) (purity ≥ 98%) were purchased from Sigma-Aldrich (St. Louis, MO, USA). Ham's F-12 (21700-075), fetal bovine serum (FBS), phosphate-buffered saline (PBS), and trypsin-EDTA solution were purchased from Gibco (Grand Island, NY, USA). 3-(4,5-Dimethythiazol-2-yl)-2,5-diphenyltetrazolium bromide (MTT), 3,3′-dihexyloxacarbocyanine iodide (DiOC_6_), and dimethyl sulfoxide (DMSO) were purchased from Sigma Chemical, Inc. (St. Louis, MO, USA). Annexin-V-FLUOS staining kit and protease inhibitor cocktail tablets were obtained from Roche Diagnostics (Rotkreuz, Switzerland). The substrates of caspase-9 (LEHD-para-nitroaniline; LEHD-p-NA), caspase-8 (IETD-para-nitroaniline; IETD-p-NA), and caspase-3 (DEVD-para-nitroaniline; DEVD-p-NA) were obtained from Invitrogen (Thermo Fisher Scientific Inc., Waltham, MA, USA).

### 2.2. Cell Culture

Human cholangiocarcinoma cell lines (KKU-100, HUCCA-1, and KKU-213) and an immortalized human cholangiocyte cell line (MMNK-1) were obtained from the Japanese Collection of Research Bioresources (JCRB) Cell Bank, Japan. All cell lines were cultured in a Ham's F-12 medium with NaHCO_3_, 100 U/mL penicillin, and streptomycin. The medium was adjusted to a pH of 7.2 and supplemented with 10% heat-inactivated fetal bovine serum. Cells were cultured at 37°C in an incubator supplied with 5% of CO_2_.

### 2.3. Cell Viability Assay

The 3-(4,5 dimethylthiazol-2yl)-2,5 diphenyltetrazolium bromide (MTT) assay [36] was performed by seeding cells in a 96-well culture plate. The stock solutions of gambogic acid (100 mM), piperine (2 M), and gemcitabine (2 M) in DMSO were used to prepare test solutions in different concentrations in Ham's F-12 medium using a 2-fold serial dilution method. The final concentration of DMSO for treatment was less than 0.1%. Cells were treated with gambogic acid, piperine, or gemcitabine (positive control) in various concentrations for a 24-hour incubation period. The cell viability in each concentration of compounds was compared to that of the untreated condition [37].

### 2.4. Determination of the Combination Index

Synergism, additivity, or antagonism between compounds was quantitated based on the Chou–Talalay method [38, 39]. The combination index (CI) value between two compounds A and B was calculated using CompuSyn Software (available by free downloading from http://www.combosyn.com) [40] employing the following equation:

(1) $$\begin{array}{c} CI=\left(\frac{C{}_{A,X}}{IC{}_{X,A}}\right)+\left(\frac{C{}_{B,X}}{IC{}_{X,B}}\right). \end{array}$$

IC_X,A_ and IC_X,B_ are concentrations of each component alone that have an *X* percent effect, whereas C_A,X_ and C_B,X_ are concentrations of compounds in combination that have the same effect. Interpretation of the value was referenced by following criteria: CI values more than 1 indicate antagonism, CI values equal to 1 indicate additivity, and CI values less than 1 indicate synergism [41, 42].

### 2.5. Apoptosis Assay

Apoptotic cell quantification was performed as previously described [43]. In brief, after compound treatment with gambogic acid and/or piperine for 24 hours, floating and adhering cells were collected and then washed with phosphate-buffered saline (PBS). After that, cells were stained with Annexin V-fluorescein isothiocyanate (FITC) and propidium iodide (PI) fluorescence dye for 15 minutes and analyzed by using a flow cytometer (CyAn ADP, Beckman Coulter, USA).

### 2.6. Determination of Mitochondrial Transmembrane Potential (ΔΨm)

This procedure was performed in accordance with the previously described method [43]. After treatment with gambogic acid and/or piperine for 24 hours, suspending and adhering cells were collected and then washed with PBS before being stained for 15 minutes at 37°C with 40 nM 3,3′-dihexyloxacarbocyanine iodide (DiOC_6_). Flow cytometry was then performed to examine the stained cells (CyAn ADP, Beckman Coulter, USA).

### 2.7. Determination of Caspases-3, -8, and -9 Activities

Caspases activity was performed according to the manufacturer's protocols by using specific substrates and colorimetric analysis. After treatment with gambogic acid and/or piperine for 24 hours, floating and adhering cells were collected and then washed with PBS. After that, the cells were lysed by using a lysis buffer and proteins were extracted. Protein extracts were incubated with caspase-3 (DEVD-p-NA), caspase-8 (IETD-p-NA), and caspase-9 (LEHD-p-NA) chromogenic substrates at 37°C for an hour. The optical density was measured by using a microplate reader (BioTek, Winooski, VT, USA) at the wavelength of 405 nm [43].

### 2.8. Statistical Analysis

All data were analyzed by using statistic SPSS Software version 20 and were presented as the mean ± standard deviation (SD) from repeated three independent experiments. Statistical analysis was performed using one-way analysis of variance (ANOVA) followed by a comparison between groups by Tukey's test when more than three groups were analyzed and using Student's *t*-test when two groups were compared. Statistically significance was considered with values of *p* < 0.05.

## 3. Results and Discussion

### 3.1. Effects of Gambogic Acid and Piperine on CCA Cell Viability

We examined the cytotoxic effect of gambogic acid and piperine on the cell viability of human CCA cell lines, including KKU-100, HuCCA-1, and KKU-213 compared to that on normal cholangiocyte MMNK-1 cells. Cells were treated with various concentrations of gambogic acid or piperine for 24 hours. We found that gambogic acid and piperine significantly inhibited viability of all CCA cells in a concentration-dependent manner (see Figure 2). Gemcitabine, a first-line drug for cholangiocarcinoma [42], was used as a positive control. Gambogic acid presented the lowest IC_50_ value in all the cancer cell lines (Table 1). However, piperine was found to be more selectively toxic, particularly against KKU-100 and HuCCA-1 cells than other compounds.

### 3.2. Piperine Enhanced the Cytotoxic Effect of Gambogic Acid against CCA Cells

To determine whether piperine could enhance the cytotoxicity of gambogic acid, CCA cells were treated with gambogic acid, piperine or in combination. The concentration of piperine was fixed at the IC_50_ value of each cell line, whereas gambogic acid concentrations ranged from 0 to 100 *μ*M. As shown in Figure 3(a), combining gambogic acid with piperine provided a synergistic anticancer effect by presenting CI values at different levels of cytotoxic effect (fraction affected, Fa) that were less than 1. However, piperine could not synergistically enhance the toxicity of gemcitabine on CCA cells (see Figure 3(b)). Interestingly, Table 2 exhibits that combination treatment of gambogic acid with piperine could reduce gambogic acid concentration when compared to a single treatment, resulting in a lower toxicity to normal cells.

### 3.3. Enhancement Effect of Piperine on Gambogic Acid-Induced Apoptotic Cell Death

Previous research has shown that gambogic acid and piperine can induce apoptosis in various cancer cells [13–15, 30]. Together with the current study, it suggested that cotreatment of gambogic acid and piperine could result in a synergistic cytotoxic effect. Hence, to elucidate the potential enhancement effect of piperine on gambogic acid-induced cell death via apoptosis, we investigated the effects of gambogic acid, piperine, and combined treatment on apoptosis in CCA cell lines. As shown in Figure 4, apoptotic cells were quantitated by Annexin V-fluorescein isothiocyanate (FITC) and propidium iodide (PI) double staining, and the result showed that the percentage of early and late apoptotic cells of combined condition was increased significantly as compared with a single treatment.

#### 3.3.1. The Combination Treatment Increased Apoptosis via Caspase Activation

To further confirm the combined effect on apoptosis induction via caspase activation, we measured caspase-3, -8, and -9 activities after treatment with gambogic acid, piperine, or a combination of two compounds for 24 hours. As shown in Figure 5, when compared to a single treatment, the activities of caspases-3, -8, and -9 increased significantly after treatment with a combination of two compounds. These results indicated that the combined treatment enhanced apoptotic cell death through both extrinsic (caspase-8) and intrinsic (caspase-9) pathways.

#### 3.3.2. The Combination of Gambogic Acid and Piperine Induced the Mitochondria-Mediated Apoptosis Pathway

Depolarization of the mitochondrial transmembrane potential (ΔΨm) as a result of mitochondrial outer membrane permeabilization (MOMP) has been shown to contribute to apoptosis induction [45, 46]. Hence, the effect of the combination treatment on the modulation of mitochondrial transmembrane potential was investigated. The mitochondrial transmembrane potential was determined by using a DiOC_6_ fluorescence probe . The results revealed that the percentage of cells with a loss of mitochondrial transmembrane potential increased significantly after treatment with a combination of two compounds when compared to a single treatment (see Figure 6).

## 4. Discussion

Because of the disease's frequent late diagnosis, chemotherapy is recommended for more than seventy percent of cholangiocarcinoma (CCA) patients [9]. However, many studies have demonstrated that there were many mechanisms of CCA cells in chemoresistance, such as reduced drug absorption and metabolism, as well as impairment of the apoptotic mechanism [47], which has resulted in a relatively poor response to existing chemotherapeutic drugs [48, 49]. Furthermore, many chemotherapeutic drugs have considerable side effects that cause patient intolerance and treatment failure. As a result, substantial efforts have been focused on finding novel and effective anticancer drugs with little or no side effects. However, the combination treatment appears to have significant potential benefits due to the reduction of side effects, the synergistic/combined antitumor effects, and the ability to overcome drug resistance [35].

Gambogic acid is the major active compound derived from *Garcinia hanburyi* [11, 12]. Previous studies have shown that it has a high efficacy anticancer effect via apoptosis induction. However, in animal studies, this compound causes many adverse effects [17–20]. One of the best options to reduce adverse reactions is cotreatment with other compounds or drugs that can enhance its activity but can reduce the toxic side effects [50]. There have been several studies that suggest a synergistic antitumor effect when gambogic acid is combined with other drugs or natural compounds [51]. Piperine, isolated from black pepper (*Piper nigrum*) and long pepper (*Piper longum*) [21], is well known as an antioxidant, antiproliferative, antiinflammatory, and anticancer agent [31, 52–55]. Moreover, it is a bioavailability enhancer for chemotherapeutic drugs and other anticancer compounds [30–32, 55]. Nevertheless, there has not been any research on its enhancement activity when combined with gambogic acid.

In the current study, the cytotoxic effects of gambogic acid and piperine were determined compared to positive control and gemcitabine. The result showed that gambogic acid, piperine, and gemcitabine inhibited the viability of cholangiocarcinoma (CCA) cells including KKU-100, HuCCA-1, and KKU213 in a concentration-dependent manner. Intriguingly, gambogic acid has the lowest IC_50_ value in all CCA cell lines. In addition, piperine was found to be more selectively toxic than the other phytochemicals (gambogic acid), especially against KKU-100 and HuCCA-1 cells. However, gemcitabine had the highest IC_50_ value and was nonselectively toxic to cancer cells.

The Chou–Talalay method was used to calculate the fractional inhibition (Fa) and combination index (CI) from the percentage of cell viability. The Fa-CI plots or the Chou–Talalay plots for drug combination in Figure 3 provide the quantitative determination of drug interactions, where CI values less than 1, equal to 1, and more than 1 indicate synergism, additive effect, and antagonism, respectively [56]. Combining gambogic acid with piperine provided a synergistic anticancer effect by presenting combination index (CI) values at different levels of the cytotoxic effect (fraction affected, Fa) that were less than 1. On the other hand, piperine could not synergistically enhance the toxicity of gemcitabine towards CCA cells. Furthermore, the combined concentrations which could inhibit CCA cell viability at 50% (IC_50_) were calculated and then were used for investigating the cell viability of normal cholangiocyte (MNNK-1). According to the synergism of piperine and gambogic acid, when compared to a single treatment, this combination decreased the concentration of gambogic acid, resulting in less toxicity to normal cells because gambogic acid exhibited nonselective toxicity, whereas piperine was found to be selectively toxic to cancer cells.

Flow cytometric analysis of apoptotic cells demonstrated that gambogic acid, piperine, and a combined treatment significantly increased the percentage of apoptotic cells compared to a single treatment. This was consistent with a significant increase in the percentage of cells with the loss of the mitochondrial transmembrane potential (ΔΨm) and the enhanced activities of caspase-3, caspase-8 (extrinsic pathway mediator), and caspase-9 (intrinsic pathway mediator) after cotreatment with gambogic acid and piperine when compared to a single treatment. These results indicated that the combination treatment synergistically inhibited CCA cell viability and was associated with apoptotic regulated cell death induction via both extrinsic and intrinsic or mitochondria-mediated pathways.

## 5. Conclusions

The purpose of this study was to demonstrate that the combination of gambogic acid and piperine synergistically suppressed cholangiocarcinoma cell (KKU-100, HuCCA-1, and KKU213) viability more efficiently than either therapy alone. Interestingly, when combined with piperine, the findings allowed the use of lower concentrations of gambogic acid in cancer treatment, perhaps reducing its adverse effect on normal cholangiocytes. In addition, the combination of the two agents enhanced apoptotic death of CCA cells through caspase and mitochondria-mediated pathways, as measured by caspase activity and the alteration of mitochondrial transmembrane potential. Taken together, the current study found that cotreatment of gambogic acid and piperine exhibited a synergistic anticancer effect on CCA cells through apoptosis induction, providing a new strategy for bile duct cancer complementary therapy. However, the mechanisms of piperine in enhancing the effects of gambogic acid should be investigated further.

## Figures and Tables

**Figure 1:** Chemical structure of (a) gambogic acid and (b) piperine.

**Figure 2:** Cytotoxic effect of gambogic acid, gemcitabine, and piperine against CCA cell lines and normal cholangiocytes. KKU-100, HuCCA-1, KKU-213, and MMNK-1 cells were treated with indicated concentrations of gambogic acid (a), gemcitabine (b), and piperine (c) for 24 h. After that, cell viability was measured using the MTT assay. Results are shown as mean ± SD values from three repeated independent experiments. In addition, ^*∗*^*p* < 0.05, ^*∗∗*^*p* < 0.01, ^*∗∗∗*^*p* < 0.001, and ^*∗∗∗∗*^*p* < 0.0001 when compared with the control (without treatment).

**Figure 3:** Combination effects of gambogic acid or gemcitabine with piperine on CCA cells. Dose-response curves (left) and CI values at different levels of fraction affected (Fa) (right) of (a) gambogic acid plus piperine and (b) gemcitabine plus piperine. Results are shown as mean ± SD values from three repeated independent experiments. In addition, ^*∗*^*p* < 0.05, ^*∗∗*^*p* < 0.01, ^*∗∗∗*^*p* < 0.001, and ^*∗∗∗∗*^*p* < 0.0001 when compared with the control.

**Figure 4:** The combination of gambogic acid and piperine significantly induced apoptosis in CCA cells. KKU-100 (a), HuCCA-1 (b), and KKU-213 (c) were treated with gambogic acid at IC_50_, piperine at IC_10_ (33.2 *μ*M, 80.7 *μ*M and 155.3 *μ*M for KKU-100, HuCCA-1, and KKU-213 cells, respectively), or combination of both for 24 hours. Then, the cells were stained with Annexin V-FITC/PI and analyzed by flow cytometry to examine apoptotic cells. Bar graphs represented the percentage of apoptotic cells. Results are shown as mean ± SD values from three repeated independent experiments. ^*∗*^*p* < 0.05 and ^*∗∗*^*p* < 0.01 compared with control (without treatment).

**Figure 5:** The combination of gambogic acid and piperine induced apoptosis via caspase activation. Caspase-3, -8, and -9 activities are shown after KKU-100 (a), HuCCA-1 (b), and KKU-231 (c) were treated with gambogic acid or piperine compared with the combined effect of the two compounds. Results are shown as mean ± SD from three repeated independent experiments. ^*∗*^*p* < 0.05 and ^*∗∗*^*p* < 0.01 compared with the control.

**Figure 6:** The combination of gambogic acid and piperine induced apoptosis via a mitochondrial pathway. After treatment, KKU-100 (a), HuCCA-1 (b), and KKU-231 (c) cells were stained with DiOC_6_ and analyzed by flow cytometry to examine the disruption of mitochondrial transmembrane potential. Bar graphs are presented as the percentage of the cells with a loss of mitochondrial transmembrane potential. Results are shown as mean ± SD, *n* = 3. ^*∗*^*p* < 0.05 and ^*∗∗*^*p* < 0.01 compared with the control.

**Table 1:** Inhibitory concentration at 50% cell viability (IC_50_) of gambogic acid, gemcitabine, and piperine on CCA cell lines compared to normal cholangiocyte (MMNK-1) and the selectivity index (SI) of each compound.

Cell type	Cell lines	Values	Gambogic acid	Piperine	Gemcitabine
CCA	KKU-100	IC_50_ (*μ*M)	63.2 ± 2.5^*∗∗∗∗*^	119.1 ± 3.6^*∗∗∗∗*^^,^^####^	1,674.7 ± 7.9
		SI	0.5	9.4	0.5
	HUCCA-1	IC_50_ (*μ*M)	53.4 ± 5.8^*∗∗∗∗*^	299.5 ± 2.4^*∗∗∗∗*^^,^^####^	1,590.1 ± 6.1
		SI	0.6	3.7	0.5
	KKU-213	IC_50_ (*μ*M)	35.7 ± 1.2^*∗∗∗∗*^	1,148.3 ± 7.3^*∗∗∗∗*^	1,423.5 ± 4.5
		SI	0.9	1.0	0.5
Normal	MMNK-1	IC_50_ (*μ*M)	31.7 ± 4.8	1,115.0 ± 6.7	768.5 ± 2.3

*Note.* The selectivity index (SI) is the IC_50_ ratio value between MMNK-1 and CCA cells. SI value less than 2 indicates general toxicity of the compound [44]. Results are shown as mean ± SD, *n* = 3. ^*∗∗∗∗*^*p* < 0.0001, significantly lower than the IC_50_ value of gemcitabine of an individual cell; ^####^*p* < 0.0001, significantly lower than the IC_50_ value of MMNK-1.

**Table 2:** Cell viability of MNNK-1 at combined concentrations which could inhibit CCA cell viability at 50% (IC_50_).

CCA cell lines	Gambogic acid (*μ*M)	Gemcitabine (*μ*M)	Piperine (*μ*M)	% cell viability of MNNK-1
KKU-100	54.9	—	157.1	77.2 ± 4.8
	—	1,482.6	157.1	53.4 ± 6.6
HUCCA-1	42.7	—	455.4	70.0 ± 2.5
	—	1,549.6	455.4	54.7 ± 3.1
KKU-213	25.7	—	1,220.1	66.6 ± 5.6
	—	1,197.2	1,206.5	47.1 ± 8.9

*Note.* The combined concentrations which could inhibit CCA cell viability at 50% were calculated using CompuSyn software.

## Data Availability

The results presented to demonstrate the findings of the current study are accessible from the corresponding author upon request.
